# Data Analysis of Educational Evaluation Using K-Means Clustering Method

**DOI:** 10.1155/2022/3762431

**Published:** 2022-07-31

**Authors:** Rui Liu

**Affiliations:** Science Teaching Department, Zhengzhou Preschool Education College, Zhengzhou 450000, China

## Abstract

It is thought to be an effective technique to handle the problem of educational data explosion and lack of information by identifying potential relationships between data and directing decision-makers through the extraction, transformation, analysis, and modeling of educational data. Based on this, this research constructs a data analysis model for education evaluation using the K-means clustering technique in DM. The weight of each index of students' comprehensive quality is calculated using AHP, and the value of the weight is used to determine whether the index is the important feature of analysis system mining. Improved sampling technology is used to deal with the representation of large-scale data sets; a sample partition clustering technique is proposed as a general framework. The best accuracy of this method, according to experimental data, is 95.6 percent, which is 12.1 percent greater than Mi cluster algorithm and 6.8 percent higher than DRCluster algorithm. The K-means clustering analysis technology is used to analyze students' comprehensive evaluation data in this paper, with the goal of determining the regularity of data implication, accurately diagnosing learning problems, and providing the foundation for developing effective student management strategies.

## 1. Introduction

With the implementation of teaching reform, enrollment continues to rise, and a large number of children face significant obstacles in terms of school construction, teaching management, and teacher management [1]. Schools have amassed a considerable amount of complex student data, such as student status information, accomplishment information, specialty information, and moral information [2]. It has been challenging to adapt the old management mode to the large student population and data management. How to properly utilize and analyze massive raw data and turn it into useable knowledge and value has become an important topic of common concern at home and abroad to tackle the difficult problems in educational data processing [3]. The introduction of information management technology to tackle data problems produced by the influx of students in the field of education has played a major role in the construction of schools [4], thanks to the rapid development of Internet technology. It is vital to acquire the necessary data for evaluating education. Researchers gradually find that the collection channels are restricted and that there are a lot of unstructured data when they collect data. It takes a long time to store meaningful data, and it is far more difficult to acquire timely information feedback [5]. Faced with these growing issues, a variety of educational applications and platforms to assist teachers in collecting and analyzing data arose and are now extensively used [6]. The rise of information technology has aided educational research by allowing for the collecting, storage, analysis, and decision-making of data and allowing for the timely collection of student studies. Simultaneously, it gives data support for teachers to properly and timely analyze students' development and change their own teaching style [7]. The introduction of information technology may not only remove a lot of repetitive manpower and increase staff efficiency, but it can also play an essential role in the collaborative administration of schools due to its fast information transmission mechanism.

DM (data mining) is also called knowledge discovery in database. DM is the process of discovering hidden, regular, and unknown but potentially useful and understandable information and knowledge from a large number of incomplete, noisy, fuzzy, and random practical application data. Cluster analysis is an important and active research field in DM [8]. As an unsupervised learning method, clustering is essentially a density estimation problem. The data to be clustered are not labeled with its category in advance and can be generated by a mixed model. Its main idea is to divide data into several classes or clusters to maximize the similarity of data objects within clusters and minimize the similarity of data objects between clusters [9]. The clustering algorithm can be selected by the data type of field attributes in the database and the characteristics of objects operated by clustering. Common clustering algorithms include partition-based clustering algorithm, hierarchical clustering algorithm, density-based method, grid-based method, model-based method, and constraint-based method. At present, large-scale data sets frequently emerge in the field of education, which poses new challenges to data analysis and research. In the face of large-scale data, traditional analysis algorithms are no longer as “handy” as small- and medium-sized data, but there are many problems such as difficult processing, long processing time, difficult parameter determination, low efficiency, and low clustering quality. Moreover, the collection content of evaluation data is single, and the analysis method lacks a certain depth. For the current situation of education data analysis, this paper introduces K-means clustering algorithm to analyze the education evaluation data. The innovations of this paper are as follows:

- From the perspective of cognitive learning theory, this paper aimed to address the current educational data's long processing time, uncertain parameters, and low clustering quality; the collection content of evaluation data is single, and the analysis method lacks certain depth and many other issues. To analyze the education evaluation data, the K-means clustering algorithm is introduced. The proposed approach is suitable for large-scale DM, according to a series of experiments. For relevant researchers, this has some reference and guiding relevance.
- In this paper, the data are cleaned, integrated, and transformed into data storage format, and the input data fulfilling the K-means algorithm are created, with the goal of solving problems such as data duplication, missing data, and inconsistent storage kinds. We may also uncover commonalities between students using the K-means technique to cluster and analyze their comprehensive evaluation results. Students are categorized based on their commonality, allowing student managers to provide tailored education management for various types of students.

## 2. Related Work

In these years of rapid DM growth, various disciplines' research topics are continually presented, including data retrieval technology, artificial intelligence, neural networks, virtual reality technology, and associated basic mathematical theories. Simultaneously, DM's applicability in the realm of education is expanding. DM has been used by a number of academics to analyze educational data in recent years.

Kelly et al. proposed a fast relaxed clustering algorithm based on graph theory. The asymptotic time complexity of this algorithm is linearly related to the data capacity when applied to larger-scale datasets [10]. Charles et al. proposed an efficient K-means clustering algorithm, which uses precomputed distances between points and dormant clusters to reduce the amount of distance computation, greatly reducing the running time and space used [11]. Rosenkranz et al. believe that the current educational data statistical analysis platforms and tools have been promoted and applied in school teaching, but there are still many problems in how to effectively analyze and use these data [12]. Scott and others believe that in the process of education, educational evaluation data occupy a large proportion, and it clearly shows the actual learning situation of students, which plays an important guiding role in teachers' teaching. Therefore, from the perspective of teachers, it uses the “Jike Big Data” system to optimize the use of educational evaluation data [13]. Hopper et al. studied the related problems of teaching optimization based on the analysis of educational evaluation data. It proposes to use educational evaluation data to determine the learning starting point of learners, design quantifiable learning goals, select learning content suitable for learners, and accurately evaluate teaching quality, and conduct personalized learning analysis and feedback in a timely manner [14]. Wolbring et al. pointed out that the collection and analysis of educational evaluation data are not only a reflection of students' learning achievements but also a reflection of teachers' teaching effect [15]. Goldberg et al. used the ideological and moral quality, intellectual education quality, physical and mental quality, and development ability quality indicators to evaluate and subdivided the indicators into multiple secondary indicators. The evaluation adopts evolutionary algorithm, fuzzy comprehensive evaluation, multivariate statistical analysis method, etc., to obtain effective weights, and the data items are summed according to the weights to obtain the quantitative score evaluation value [16]. Kang et al. selected some data from a large-scale data set, used these data to construct an adjacency matrix, and obtained eigenvectors by eigendecomposition of the adjacency matrix, and finally used Nyström to approximate the eigensolution of the original matrix [17]. Aiming at the main methods of DM, Hou et al. studied the ideas and applications of related algorithms, analyzed the advantages and disadvantages of existing methods and compared them. Based on this, a data analysis method based on the optimal decision tree algorithm is proposed [18]. Lavelle et al. analyzed and designed an evaluation database based on the functional requirements of the school education and teaching situation evaluation system. It can realize functions such as maintenance of basic information, statistics, and query of evaluation data [19]. Wang et al. proposed a new fuzzy clustering algorithm based on genetic algorithm, which realized the clustering analysis of characteristic data with mixed attributes. By introducing the genetic algorithm into the algorithm, the global optimal solution can be obtained quickly and effectively, and it does not depend on prototype initialization at all [20].

Based on these studies, this paper proposes an educational evaluation data analysis method based on K-means clustering algorithm to solve the problems of difficult processing, long processing time, and difficult parameter determination. In this paper, firstly, the cluster analysis method in DM technology is applied to establish a model to quantitatively analyze the indicators and their values of objects, and then, a new comprehensive evaluation method for students combining quantitative analysis with qualitative analysis is proposed. Then, AHP is used to calculate the weight of each index of students' comprehensive quality and judge whether the index is the key attribute of analysis system mining according to the value of the weight. Finally, the improved sampling technique is used to deal with the representation of large-scale data sets. A general framework of sampling partition clustering algorithm is proposed. The validity of the framework is verified by implementing K-means and k-medoids algorithms. It is proven that this method is practical and feasible.

## 3. Methodology

### 3.1. DM-Related Technology

With the gradual development of educational big data, artificial intelligence, learning analysis, and intelligent network learning platform, learners' whole-process learning data can be recorded. At the same time, with the rapid development of DM, artificial intelligence, and other technologies, these educational data can be automatically and deeply analyzed and processed, and learners can be personalized analyzed and diagnosed. The core function of DM technology is to discover potential rules from large-scale data. DM (data mining) is a specialized technology for mining extraordinary knowledge from large-scale data. It is a process of mining useful information from incomplete, massive, noisy, fuzzy, and random data that people do not know in advance. DM is a process of discovering potentially useful information or knowledge in reality. This process is essential for discovering knowledge in the database, in which knowledge discovery is a process of converting raw data into effective information that can be used for analysis. DM is a process of selecting, exploring, and modeling a large amount of data to discover unknown rules and relationships in advance. The purpose of DM is to get clear and useful results for the owner of education database. The DM process generally consists of business object determination, data preparation, DM, and result analysis.

Cluster analysis in DM is an active and challenging research field. In recent decades, its importance and cross characteristics with other research directions have been widely recognized by people. It plays a very important role in identifying the internal structure of data and has become one of the important research contents of DM, machine learning, and pattern recognition. The differences between groups are obvious, and the data in the same group are as similar as possible. Data clustering divides physical or abstract objects into several groups. Within each group, there is high similarity between objects, but low similarity between groups. It is the same as and different from classification. The same thing is that the data source is divided into several parts. The difference is that it is a kind of unsupervised learning, and it does not know the final grouping number and grouping standard. As a classical clustering algorithm, K-means mainly realizes different classifications of data sets through an iterative process. This algorithm has the advantages of simplicity and strong scalability. In DM field, the typical requirements for clustering mainly include the following aspects: ① scalability, ② ability to handle attributes of different data types, ③ any shape cluster can be found, ④ insensitive to the entered record order, ⑤ high dimension, ⑥ minimization of domain knowledge for determining input parameters, ⑦ ability to effectively deal with noise and abnormal data, and ⑧ availability and interpretability. In DM stage, the task or goal of mining is determined, and the mining method is selected, to implement DM operation and obtain useful patterns. The specific DM application requirements are determined, the goal of mining is cleared, and the effect that can be achieved after the system is completed. The application field background is analyzed, and the problem objective is determined. The background knowledge of related fields is understood, the needs of users are made clear, and data are collected to solve problems, and services are provided for the follow-up work. Traditional data analysis is a kind of verification analysis. It is a kind of user-driven data analysis, focusing on describing the facts that have happened in the past. DM is to mine information and discover knowledge without hypothesis. The obtained information has three characteristics: effective, unknown in advance, and practical. It is to predict the future situation and explain the factual reasons of the past. To obtain potentially effective information to meet the needs of users, it is required to fully mine the surface information, remove redundant data, and visually display key data to users. Prediction and description are the two goals of DM. Prediction refers to the use of some information fields and variables in the database to predict the hidden useful information, and description refers to the description of data as an understandable pattern. There are two aspects to consider when choosing an algorithm: first, according to the different characteristics of different data, the algorithm is selected related to it to mine; second, according to the needs of users or the actual operation of the system. This stage is the core and difficulty of knowledge discovery process.

### 3.2. Big Data of Education and Educational Evaluation

This paper holds that educational big data refer to the data collection generated in the whole process of educational activities and collected according to educational needs, which is used for educational development and can create great potential value. Big data for education are a subset of big data, and it is a collection of data generated throughout the educational process and collected based on educational needs, which is utilized for educational improvement and has a lot of potential value. Schools have purchased or adapted educational administration systems to better handle students' information as the student population has grown. The system's principal purpose is to keep track of pertinent information about pupils' academic achievement, for example, students' test scores and grade points, information about their curriculum, examination schedules, attendance, and information regarding rewards and discipline violations, among other things. All of this is educational big data. Different classification standards exist for big education data, depending on the perspective. Teaching data, management data, scientific research data, and service data can all be found in the data sources. According to the degree of organization, it can be separated into structured data, semi-structured data, and unstructured data. It can be separated into process data and result data at the collection stage. Process data are information gathered during the teaching process that is difficult to quantify directly. Quantifiable data are referred to as result data.

A huge education database is built to collect massive student data, including students' test scores, social activities, class attendance, and hobbies. Relying on tens of millions of data collected by the database can help students in various universities to do data analysis, help them find out the reasons why they cannot improve their grades, and help them adjust their learning styles or change their lifestyles in time to avoid dropping out of school. The data collected in each evaluation are defined as educational evaluation data in this paper, and the data types are mainly data generated in the learning process including the knowledge points, questions, difficulty, discrimination, learners' right and wrong situation, grades, and ranking. At present, the application value of educational evaluation data is mainly reflected in six aspects, namely, promoting more scientific teaching management, promoting the innovation and reform of teaching mode, promoting the realization of personalized learning, promoting the reconstruction of educational evaluation system, promoting the successful transformation of scientific research paradigm, and promoting the humanization of educational service. Educational evaluation refers to the process of scientifically measuring and judging various educational activities, educational processes, and educational results using certain technologies and methods under the guidance of certain educational values and according to established educational goals. At present, the research in the field of basic education has just started, and the data analysis platform of education evaluation has not been able to provide accurate education decisions for teachers and personalized teaching services for students. Therefore, the research on educational big data needs to be strengthened.  Figure 1 is a teaching optimization method based on educational evaluation data.

Education evaluation data are the data fact obtained for the education effect or the development of students in all aspects, and education evaluation is the process of value judgment based on these data. Student evaluation data are one of the subsets of educational big data that educators are most familiar with. Its sources are abundant, including formative evaluation, unit test, midterm and final test, and large-scale regional test. There are various types of data, including test scores and teacher evaluation. When confronted with diverse and customized student groups, fixed, homogenous, and dogmatic educational and administrative systems have revealed numerous flaws. To reform educational techniques and management modes, we should begin with the dominant position of students and provide tailored instruction based on their qualities. In school education, evaluation data are regarded as the most important indicator of educational and teaching improvement. These data are mainly test scores gathered through measurement, and careful collection, categorization, sorting, statistics, and analysis can turn them into very valuable big data in education. Teachers are the leaders of pupils in the sphere of education. The more they know about students, the better they can choose the most appropriate learning content in class, set the most precise learning objectives, conduct objective learning evaluations and provide timely learning feedback, provide students with personalized guidance, and help them develop their abilities to their full potential. The use of educational evaluation data analysis software or tools in the teaching process, as well as the routine collecting and analysis of these data, is critical to maximizing the value of evaluation data. Teachers can stay on top of changes in their students' knowledge, help them modify their learning speed, and continually enhance and optimize the instructional design process.

### 3.3. Educational Evaluation Data Analysis Based on K-Means Algorithm

Data integration, data selection, and data preprocessing are the three sub-steps of data preparation. Data integration unifies data from numerous files or databases, cleans it, and resolves semantic ambiguity. The goal of data selection is to figure out what the operation object of the discovery task is, which is the target data, which is a collection of data taken from the original database to meet the demands of users. The goal of data preparation is to convert raw data into a format that can be analyzed. Data preprocessing entails combining data from several sources, eliminating duplicate data values and noisy data, and screening out data sets and feature qualities that are not relevant to present DM activities. K-Means uses the rule algorithm to compute the distance between data items and then iteratively calculates the grouping situation of the obtained data objects until the center does not move, resulting in K clustering outcomes. The general algorithm flow is shown in Figure 2.

After the DM stage, the obtained result patterns are usually redundant or do not meet the user's requirements, so it is necessary to delete, filter, or return to the previous stage according to certain standards and reselect data and methods to obtain meaningful patterns and knowledge. In the course of the task, different data sources and different formats of the collected data are also different, so different data should be integrated and cleaned and processed. The general process of clustering includes feature selection, similarity measurement, clustering algorithm, result verification, and decision-making. K-Means algorithm is simple and efficient. However, there is no clear standard definition for the clustering number *k* and the selection of the center point of the algorithm, and most of them are given randomly, which will easily cause great influence on the algorithm results. Therefore, a selection method to solve the initial value *k* is used. Given a set of *n* data points:

(1) $$\begin{array}{c} X=\left\{x_{1},x_{2},x_{3},\ldots ,x_{n}\right\}. \end{array}$$

The algorithm is to find a partition of *X*, *P*_*k*_={*C*_1_, *C*_2_, *C*_3_,…, *C*_*k*_}, which minimizes the value of the objective function *J*.

(2) $$\begin{array}{c} J={\sum_{i=1}^{k}\sum_{x_{j}\in C_{i}}\left|x_{j}-o_{i}\right|}^{2}, \end{array}$$

where *o*_*i*_ represents the center point of class *C*_*i*_. The Euclidean distance between two *p*-dimensional data points *x*_*i*_ and *x*_*j*_ is set, as in formula:

(3) $$\begin{array}{c} x_{i}=\left(x_{i1},x_{i2},x_{i3},\ldots ,x_{ip}\right),\\ x_{j}=\left(x_{j1},x_{j2},x_{j3},\ldots ,x_{jp}\right),\\ d\left(x_{i},x_{j}\right)=\sqrt{{\left(x_{i1}-x_{j1}\right)}^{2}+{\left(x_{i2}-x_{j2}\right)}^{2}+\ldots +{\left(x_{ip}-x_{jp}\right)}^{2}}. \end{array}$$

The average distance of all samples is determined as follows:

(4) $$\begin{array}{c} \text{Meandist}\left(S\right)=\frac{2}{n\left(n-1\right)}\times \sum_{i\neq j,i,j=1}^{n}d\left(x_{i},x_{j}\right). \end{array}$$

The square error criterion function for determining the objective function is as follows:

(5) $$\begin{array}{c} \sigma_{i}=\sqrt{\frac{{\sum_{i=1}^{n_{i}}\left(x_{i}-c_{i}\right)}^{2}}{C_{i}-1}}. \end{array}$$

In the formula, *c*_*i*_ is the centroid point of the same category of data. The *c*_*i*_ calculation formula is defined as follows:

(6) $$\begin{array}{c} c_{i}=\frac{1}{\left|C_{i}\right|}\sum_{x_{i}\in T_{i}}x_{j}. \end{array}$$

In the formula, |*C*_*i*_| is the number of *C*_*i*_-like data objects; *c*_*i*_ represents the *i*th cluster center.

Data cleaning is the process of cleaning problematic data. Its task is to clean the data that do not meet the requirements, usually deleting or modifying, but not simply modifying. Data that do not meet the requirements are redundant, missing, and wrong data. Data cleaning mainly includes standardization of format, removal of abnormal data and duplicate data, and correction of error data. It is necessary to clear some duplicate data in the test data management system and obtain data of other dimensions from other systems to supplement the whole database. The purpose of data cleaning is to ensure the accuracy and validity of data, to ensure good mining efficiency in the process of mining. At the same time, data cleaning is the foundation to complete the whole mining work. Given data input as information, features are extracted to represent the whole data set, so that redundant information can be reduced as much as possible. Then, according to the similarity between data points, a specific clustering algorithm is applied to the data set, and the cost function usually determined by the similarity of data points is reduced to the minimum. When the algorithm converges, it will return the output cluster. Clustering is very complicated. Different clustering analysis is applied to the same data, and the results are completely different, and the definition of clustering is usually relative. There are different clustering methods for the same group of objects, and different clustering of the same data probably corresponds to different applications.

Based on the minimum distance principle, we classify the data points *x* in the remaining datasets into the current cluster, namely,

(7) $$\begin{array}{c} c=\arg\min\left({\left|x-\mu_{j}\right|}^{2}\right), \end{array}$$

where *μ*_*j*_ is the centroid of class *C*_*j*_ and *c* is the class assigned to the data. Once new data have been assigned a class label, the cluster centroids are updated iteratively until all data points have been processed:

(8) $$\begin{array}{c} \mu_{j}=\frac{\mu_{j}m_{j}+x}{m_{j}+1},m_{j}=m_{j}+1. \end{array}$$

The data in the assessment system can be separated into two groups: one that can be represented using mathematical language and another that can be stated using words. The language's data can be examined and sorted, and DM technology's decision tree, correlation analysis, and cluster analysis methods can be used to create a model to quantify the analysis object. Because of the irregularity of data acquired from various sources, data conversion is required to develop a process suitable for DM. The quality of K-means clustering is insecure when dealing with huge data sets. As a result, this study introduces a sampling strategy to make the partition clustering algorithm acceptable for large-scale data sets. The simplest way is to choose numerous partitions at random from the original large-scale data collection. Each partition employs a clustering technique, with clustering results that are both reliable and capable of representing the entire data set. Input data are information saved on various digital media in various formats, such as an electronic report or a data relation table. These data might be kept in centralized databases or distributed site systems.

## 4. Result Analysis and Discussion

This study investigates the impact of data analysis on education evaluation using the K-means algorithm, as well as conducting teaching trials. The similarities between students are discovered through clustering analysis of students' comprehensive evaluation scores using the K-means technique. Students are categorized based on their commonality, allowing student managers to provide tailored education management for various types of students. The evaluation findings and learners' understanding levels are assessed before and after deployment, and the learning effect provided by this model is tracked. During the experiment, learners were interviewed and given questionnaires to gain feedback and suggestions for optimizing and refining the model, which was then iteratively improved to measure its overall performance. Finally, a feedback questionnaire is created to assess the model's use feedback across several dimensions. To begin, this section compares and contrasts the efficiency and effect of the DRCluster and Mi cluster algorithms with this algorithm, as well as analyzes and evaluates their biological importance. The running efficiency of different algorithms is shown in Figure 3. The accuracy of different algorithms is shown in Figure 4.

It can be seen that the running efficiency of this algorithm is high, and the running efficiency of DRCluster algorithm and Mi cluster algorithm is lower than that of this algorithm. In terms of recall rate, this method also has certain advantages, and the recall rate of this method is better than the other two algorithms. This conclusion also verifies the superior performance of this algorithm. To further evaluate the mining effectiveness of the algorithm, different algorithms are used for biclustering mining of six data sets, and the number of biclusters they can find is compared.  Table 1 shows the number of double clusters that the three algorithms can mine in six data sets.

It can be seen from the table that the Mi cluster algorithm can find the least number of double clusters, which is mainly related to the differential support defined by the algorithm. However, the algorithm in this paper adopts effective support degree, transformation into differential weight graph, effective pruning strategy, and so on, which makes the number of mining biclusters the largest. A significant amount of experimental data are analyzed in this section. The software Office Visio was used to create the expert knowledge structure map and the student knowledge structure map. The Questionnaire website was used to gather and evaluate student feedback questionnaires, which were then analyzed using SPSS. The educational administration employees should compile the basic data needed for the evaluation and keep track of pertinent information such as the classes participating in the evaluation, the class teachers, the class subjects, and the teachers prior to the evaluation. Second, a system is set for students to rate their teachers and classmates. Finally, the evaluation is questioned by leaders and teachers. The analysis and application of educational evaluation data will examine every student's homework, test, and examination, transforming diagnostic evaluation into process evaluation and allowing teachers to grasp students' learning progress and place in time and reflect and adjust their teaching accordingly. Figures 5 and 6 depict the outcomes of clustering data sets using the DRCluster algorithm, Mi cluster algorithm, and this algorithm mode, respectively.

The test results reveal that the suggested method has a high level of accuracy, with an error rate of less than 2% over time. In these three modes, the K-means clustering algorithm suggested in this paper is valid. Routine exercises and examination evaluation tasks are carried out by students. Explicit data are the result of statistically studied evaluation data, such as score ranking, true or false situations, and answer time. Qualitative outcomes that require more examination, such as knowledge structure and comprehension level, are referred to as implicit data. The thorough evaluation score sheet includes factors such as ideological quality, cultural and athletic activity innovation, and academic accomplishment. All scores are in percentages, with a minimum scoring unit of 1 and no order of magnitude difference. The existing data dimension table is separated into three categories, and the values are taken according to the supplied weight coefficient, to compare with the current measurement and quantification result data. Students' evaluation data collection uses marking instrument and extreme class big data platform, and teachers use extreme class big data platform to arrange knowledge unit test papers, print them into papers, and distribute them to students. The test paper scanner is used to collect students' evaluation data, and the students' evaluation data are stored in the polar class big data platform. The evaluation data are analyzed, and the achievement of learning goal A of a class after the implementation of targeted education management is analyzed as shown in Table 2.

It can be seen that the total success rate of the class is 92.14%. The overall average score rate of the class is higher than that of the grade, which indicates that the class has a good grasp. Using K-means algorithm, DRCluster algorithm, and Mi cluster algorithm, the comprehensive evaluation scores of students are clustered and analyzed, respectively, and then, the changes in students' test scores after implementing targeted education management for different types of students are shown in Figure 7.

From the data analysis in Figure 7, it can be seen that after the analysis and targeted teaching management with this method, the students' scores show an obvious upward trend. Its influence on the improvement of students' grades is far greater than the other two methods. This result shows that this method is effective and feasible.

## 5. Conclusions

E-learning institutions contain a lot of useful information. Many educators are grappling with how to accurately uncover the important knowledge concealed in school evaluation data in the midst of such a massive amount of data. This work creates an educational evaluation data analysis model based on the K-means clustering method from the perspective of cognitive learning theory, based on existing research and application of educational evaluation data analysis at home and abroad. The model generates corresponding categorization rules based on a large number of students' educational assessment data; the main factors that can affect students' overall quality are determined based on the study of these rules. In addition, the K-means clustering algorithm is used to statistically assess the indicators and their values of the objects, resulting in the proposal of a new comprehensive student evaluation technique that combines quantitative and qualitative analysis. Experiments demonstrate that this method can achieve a maximum accuracy of 95.6 percent, which is 12.1 percent higher than Mi cluster and 6.8 percent higher than DRCluster. This method efficiently solves the drawbacks that traditional algorithms have, such as low processing per unit time, high processing times when dealing with big amounts of data, and difficulty in attaining the desired results. It has some practical and theoretical value in the field of data analysis, as well as some reference value for other academics. Despite the fact that this study accomplished certain research outcomes, numerous influencing factors and controls were not taken into account in the design process due to time constraints and a lack of understanding. The analysis technique will be improved in the future to improve the educational evaluation data analysis model. [21].

## Figures and Tables

**Figure 1:** Teaching optimization method based on educational evaluation data.

**Figure 2:** General flow of K-means clustering algorithm.

**Figure 3:** Running efficiency of different algorithms.

**Figure 4:** Recall of different algorithms.

**Figure 5:** Accurate recognition rate.

**Figure 6:** False recognition rate.

**Figure 7:** Changes in student achievement.

**Table 1:** Comparison of algorithm effectiveness.

Data set	Number of genes	Number of samples	Mi cluster algorithm/number of biclusters	DRCluster algorithm/number of double clusters	Number of algorithms/biclusters in this paper
Yeast	21498	297	30	139	254
Lymphoma	11024	209	37	131	167
Breast	3014	184	42	126	326
Live	4125	99	51	154	312
Lung	54926	82	15	142	106
Path_ metabolic	801	73	9	136	89

**Table 2:** Analysis of the achievement of students' learning objective A.

Student number	Students should meet the standards	Actual score rate of students	Determine whether students meet the standard	Class should meet the standard (%)	Actual score rate of class (%)	Actual grade score rate (%)	Probability of reaching the standard (%)
1	72%	80%	Yes	80.57	92.75	88.69	92.14
2	75%	90%	Yes				
3	88%	100%	Yes				
4	90%	95%	Yes				
5	93%	100%	Yes				
6	96%	100%	Yes				
…	…	…	…				

## Data Availability

The data used to support the findings of this study are included within the article.

## References

[1] Jan M. A. (2021). *Application of Big Data, Blockchain, and Internet of Things for Education Informatization*.

[2] Hall W. A. (2013). Consumerism and consumer complexity: implications for university teaching and teaching evaluation. *Nurse Education Today*.

[3] Weston T. J., Hayward C. N., Laursen S. L. (2021). When seeing is believing: generalizability and decision studies for observational data in evaluation and research on teaching. *American Journal of Evaluation*.

[4] Antoci A., Brunetti I., Sacco P., Sodini M. (2020). Student evaluation of teaching, social influence dynamics, and teachers’ choices: an evolutionary model. *Journal of Evolutionary Economics*.

[5] Sánchez T., Gilar-Corbi R., Castejón J. L., Vidal J., Leon J. (2020). Students’ evaluation of teaching and their academic achievement in a higher education institution of Ecuador. *Frontiers in Psychology*.

[6] Johnson M. D., Narayanan A., Sawaya W. J. (2013). Effects of course and instructor characteristics on student evaluation of teaching across a college of engineering. *Journal of Engineering Education*.

[7] Prochazkova K., Novotny P., Hancarova M., Prchalova D., Sedlacek Z (2019). Teaching a difficult topic using a problem-based concept resembling a computer game: development and evaluation of an e-learning application for medical molecular genetics. *BMC Medical Education*.

[8] Bergin C., Wind S. A., Grajeda S., Tsai C. L. (2017). Teacher evaluation: are principals’ classroom observations accurate at the conclusion of training?. *Studies In Educational Evaluation*.

[9] Litke E., Boston M., Walkowiak T. A. (2021). Affordances and constraints of mathematics-specific observation frameworks and general elements of teaching quality. *Studies In Educational Evaluation*.

[10] Kelly M., Bennett D., Mcdonald P. (2012). Evaluation of clinical teaching in general practice using the Maastricht Clinical Teaching Questionnaire. *Medical Teacher*.

[11] Charles E. G. (2016). The teaching model and evaluation of teaching performance. *The Journal of Higher Education*.

[12] Rosenkranz S. K., Wang S., Hu W. (2015). Motivating medical students to do research: a mixed methods study using Self-Determination Theory. *BMC Medical Education*.

[13] Scott K. M., Baur L., Barrett J. (2017). Evidence-based principles for using technology-enhanced learning in the continuing professional development of health professionals. *Journal of Continuing Education in the Health Professions*.

[14] Hopper M. K. (2016). Assessment and comparison of student engagement in a variety of physiology courses. *Advances in Physiology Education*.

[15] Wolbring T., Treischl E. (2016). Selection bias in students’ evaluation of teaching. *Research in Higher Education*.

[16] Goldberg D. E., Somerville M. (2015). The making of*A whole new engineer*: four unexpected lessons for engineering educators and education researchers. *Journal of Engineering Education*.

[17] Kang M. J., Ngissah R. K. S. (2020). Self-reported confidence and perceived training needs of surgical interns at a regional hospital in Ghana: a questionnaire survey. *BMC Medical Education*.

[18] Hou Y. W., Che-Wei L., Gunzenhauser M. G. (2017). Student evaluation of teaching as a disciplinary mechanism: a foucauldian analysis. *The Review of Higher Education*.

[19] LaVelle J. M. (2018). Book review: building evaluation capacity: activities for teaching and training. *American Journal of Evaluation*.

[20] Wang W. (2021). Evaluation principles’ influence of critical thinking foreign language teaching on German literature classroom learning motivation. *Revista de Cercetare şi Intervenţie Socială*.

[21] Sendra-Portero F., Torales-Chaparro O. E., Ruiz-Gómez M. J., Martinez-Morillo M (2013). A pilot study to evaluate the use of virtual lectures for undergraduate radiology teaching. *European Journal of Radiology*.

